RETRACTED

# Seed germination ecology of *Conyza sumatrensis* populations stemming from different habitats and implications for management

**DOI:** 10.1371/journal.pone.0260674

**Published:** 2021-12-02

**Authors:** Yanyun Xu, Junyong Ye, Ahlam Khalofah, Ali Tan Kee Zuan, Rehmat Ullah, Ahmed M. El-Shehawi

**Affiliations:** 1 College of Ecology, Lishui University, Lishui, China; 2 Rural Industry Development Center of Liandu District, Lishui, China; 3 Department of Biology, Faculty of Science, King Khalid University, Abha, Saudi Arabia; 4 Research Center for Advanced Materials Science (RCAMS), King Khalid University, Abha, Kingdom of Saudi Arabia; 5 Department of Land Management, Faculty of Agriculture, Universiti Putra Malaysia, Selangor, Malaysia; 6 Soil and Water Testing Laboratory for Research, Dera Ghazi Khan, Punjab, Pakistan; 7 Department of Biotechnology, College of Science, Taif University, Taif, Saudi Arabia; Harran Üniversitesi: Harran Universitesi, TURKEY

## Abstract

*Conyza sumatrensis* (Retz.) E. H. Walker is an obnoxious weed, emerging as an invasive species globally. Seed germination biology of four populations of the species stemming from arid, semi-arid, temperate, and humid regions was determined in this study. Seed germination was recorded under six different environmental cues (i.e., light/dark periods, constant and alternating day and night temperatures, pH, salinity, and osmotic potential levels) in separate experiment for each cue. Populations were main factor, whereas levels of each environmental cue were considered as sub-factor. The impact of seed burial depths on seedling emergence was inferred in a greenhouse pot experiment. Seed germination was recorded daily and four germination indices, i.e., seed germination percentage, mean germination time, time to reach 50% germination, and mean daily germination were computed. Tested populations and levels of different environmental cues had significant impact on various seed germination indices. Overall, seeds stemming from arid and semi-arid regions had higher seed germination potential under stressful and benign environmental conditions compared to temperate and humid populations. Seed of all populations required a definite light period for germination and 12 hours alternating light and dark period resulted in the highest seed germination. Seed germination of all populations occurred under 5–30°C constant and all tested alternate day and night temperatures. However, the highest seed germination was recorded under 20°C. Seeds of arid and semi-arid populations exhibited higher germination under increased temperature, salinity and osmotic potential levels indicating that maternal environment strongly affected germination traits of the tested populations. The highest seed germination of the tested populations was noted under neutral pH, while higher and lower pH than neutral had negative impact on seed germination. Arid and semi-arid populations exhibited higher seed germination under increased pH compared to temperate and humid populations. Seed burial depth had a significant effect on the seedling emergence of all tested populations. An initial increase was noted in seedling emergence percentage with increasing soil depth. However, a steep decline was recorded after 2 cm seed burial depth. These results indicate that maternal environment strongly mediates germination traits of different populations. Lower emergence from >4 cm seed burial depth warrants that deep burial of seeds and subsequent zero or minimum soil disturbance could aid the management of the species in agricultural habitats. However, management strategies should be developed for other habitats to halt the spread of the species.

RETRACTED

## Introduction

*Conyza sumatrensis* had been known as *Erigeron sumatrensis* and *Conyza albida* Wild. ex. sprang. until 1971; afterwards, it was named as *C*. *sumatrensis* [1, 2]. It is a tall broad-leaved fleabane [3] and belongs to Asteraceae family. It is broad-leaved, seed-reproducing, annual or biennial, herbaceous species [3, 4]. The stem of *C*. *sumatrensis* branches upward and forms a flower head. Although a plant of the species is usually 100–200 cm in height, it can reach to 3 m height. The stem is green, hairy, round, upright, angular, and striped. The trunk is branched, upward with many leaves and resembles a pine tree in appearance. The lateral branches are shorter than the main stem and densely hairy. Basal leaves are in rosette form and can be straight or toothed. Leaves are grayish green, the edges are hairy, and the leaves are in an upright position. The leaves are alternate and lack petiole. The leaf blade is round, 10 cm long and 1.5 cm wide. Leaf margins are generally toothed, lower leaves have more prominent teeth than upper ones and are sparsely hairy. The flower has a disc structure and is 4–10 mm in diameter when dry. Numerous flowers are formed at the top of the plant, at the tip of the stem. The flowers are white or light yellow. Sepals are dark and pale in color, sometimes with pink stripes. It is approximately 3 rows of narrow, round, sparsely hairy, thin pointed and tubular structure [5].

It is considered as a noxious weed of several cropping systems around the world [6, 7]. It is observed between lower altitudes. The species is also used in different folk medicines in various cultures [8]. Ongoing climate changes have transitioned conventional agricultural practices to conservational practices [9, 10] due to which new weed species have been observed and increasingly becoming difficult to manage [7, 11, 12]. Nonetheless, influence of different environmental cues on seed germination of different populations of the species is also unknown. The missing knowledge of seed germination of these species is a hurdle in their management. Seed germination of weed species could be halted by creating unsuitable environmental conditions [13–16]. Recently Mahajan et al. [17] studied seed germination biology of two populations (herbicide resistant and susceptible) of *C*. *sumatrensis* stemming from Australia under various environmental cures. The authors reported significant differences among the populations and warned that herbicide resistant population could invade more area due to its higher germination ability under a broad range of temperatures. Similarly, Ali et al. [18] studied seed germination biology of *C*. *stricta* and reported that the species had the potential to extend its range; thus, immediate management strategies are needed for different habitats to halt the further spread of the species. However, seed germination biology of *C*. *sumatrensis* populations stemming from different climatic regions remains unknown.

RETRACTED

Several environmental cues exert significant impacts on seed germination and seedling emergence of weeds and crop plants [19–22]. These environmental cues include temperature, light/dark period, abiotic stresses, soil pH and seed burial depth [13–16]. Light has a positive impact on the seed germination of almost all *Conyza* species which require a definite light period for their successful seed germination [18, 23, 24]. Moreover, seeds of these species buried deep in the soil are unable to emerge due to unavailability of sufficient light for completing germination phase [13, 15, 25–27]. Seed germination of weed species is strongly impacted by the presence/absence of seed dormancy. Nevertheless, seed dormancy is important for weed species for longer persistence in the soil seed bank. Low or no seed dormancy is observed in *Conyza* species [28], although some reports indicated that these species are highly dormant [29]. Like all other weed species, seeds of *Conyza* species undergo dormancy under stressful environments and resume germination once environmental cues are favorable [30].

Several enzymes necessary for seed germination are regulated by temperature; thus, it is an important environmental cue influencing seed germination of weeds and crop plants [31]. *Conyza* species successfully germanite under a temperature range of 20 and 30°C, and 20°C is regarded optimum for their seed germination [23, 26–28, 32, 33]. Nonetheless, some studies have reported that several *Conyza* species are capable of germinating at higher temperatures [24, 26, 32]. Due to the reason, inferring seed germination of each species under various environmental cues is necessary for their successful management.

RETRACTED

*Conyza* seeds require definite light period for their seed germination; thus, emerge from the upper soil layers [26, 30]. Absence of seed dormancy in *Conyza* species is a big hurdle in their longevity in the soil seed bank [28]. Nevertheless, these species can produce huge amounts of seeds and seed production enables their spread and invasion. Higher seed production results in more number of seedlings emerging per unit area; thus, the species can stay in different cropping systems [34]. Determining seed germination biology and inferring the impact of seed burial depth on seedling emergence would aid in the development of management options for weed species [35, 36]. However, such knowledge is not available for *C*. *sumatrenis*. Therefore, current study determined the impact of different environmental cues on seed germination and seedling emergence of four population of *C*. *sumatrenis* arising from arid, semi-arid, temperate, and humid regions. It was hypothesized that tested populations will have varying seed germination due to maternal environments. The knowledge of seed germination biology will help to manage the species in the existing cropping systems.

## Materials and methods

### Seed collection

Seeds from different established populations in arid, semi-arid, temperate, and humid climatic regions were collected from randomly selected 100 plants (Table 1). Seeds were collected from established populations for at least five years to have the maternal effects transferred. Soil characteristics of the seed collection sites are given in Table 1. Seed present on fifty mother plants were collected and used in the experiments. Since *C*. *sumatrensis* is not an endangered species and not regulated by any quarantine laws, study was exempt from permits.

**Table 1:** Physical and chemical characteristics of the soils in different climatic regions of seed collection sites.

Habitat	Latitude °N	Longitude °E	CaCO_3_ (%)	OM (%)	pH	EC (mS/m)	Clay (%)	Sand (%)	Silt (%)	P (ppm)
Semi-arid	30.422621	72.346786	43.00	0.34	8.11	387.89	47.70	27.30	25.00	49.35
Temperate	33.727609	73.133604	32.12	0.68	7.34	101.30	28.20	46.30	25.50	33.18
Humid	28.101736	69.662429	33.45	1.12	7.45	94.12	41.70	25.30	27.00	45.76
Arid	30.954379	70.932017	45.67	0.89	8.34	470.13	33.10	45.40	21.50	33.22

OM = organic matter, P = phosphorus, EC = electrical conductivity.

RETRACTED

### Experimental details

Seven different experiments (each comprising of one environmental cue and its different levels) were conducted to infer the germination ability of the seeds collected from four populations in varying climatic regions (Table 1). The information regarding different environmental cues and their levels used to determine seed germination of different populations are given in Table 2. Seeds were non-dormant; therefore, freshly harvested seeds were used in the study. Chauhan et al. [37] and Michel and Kaufmann [38], were followed to prepare the solutions of desired salinity stress and osmotic stress levels, respectively.

**Table 2:** Different environmental cues and their levels used to study seed germination biology of *Conyza sumatrensis* populations collected from varying climatic regions.

Environmental cues	Treatments
Light/dark duration (hours)	0, 12, 24
Constant temperature (°C)	5, 10, 15, 20, 25, 30, 35, 40
Fluctuating day/night temperature (°C)	15/10, 20/15, 15/15, 20/10
Salinity stress treatments (mM NaCl)	0, 25, 50, 100, 150, 200, 250, 300, 350, 400, 450, 500
Osmotic stress levels (-MPa)	0, 0.1, 0.2, 0.3, 0.4, 0.5, 0.6, 0.7, 0.8, 0.9, 1.0
pH levels	3, 4, 5, 6, 7, 8, 9, 10,
Seed burial depths (cm)	0, 1, 2, 3, 4, 5, 6, 7, 8

### Experimental design

Factorial design was followed to conduct the experiments on seed germination and seedling emergence. The populations were considered as main factor, whereas levels of the tested environmental cues were regarded as sub-factor. The experiments were separate for each environmental cue. All experiments were repeated over time to validate the results.

### Experimental procedure

Petri-dish laboratory experiments were conducted to observe the germination of seeds collected from various climatic regions, whereas a pot experiment was conducted to infer seedling emergence from different seed burial depths. Petri dishes were sterilized before the initiation of the experiments to avoid any contamination and fungal attack. The round discs of Whatman no. 1 filter paper were fixed in the Petri dishes upon which seeds were places and treatment solutions were applied. Each dish had 60 seeds to observe the germination. The dishes were provided with 5 ml of solutions of various treatments and sealed with paraffin film. Afterwards, the dishes were placed at respective environmental conditions. Generally, seed germination was observed under 20/15°C day/night temperature. However, Petri dishes in constant and fluctuating day/night temperature experiment were placed at their relevant temperatures. The experiment lasted for 3 weeks, and germinating seeds were counted daily. Seed germination and seedling emergence percentage was computed from the number of germinated/emerged seeds and used for the interpretation of the results. Three different seed germination indices, i.e., mean germination time, time to reach 50% germination and mean daily germination were computed by using Eqs 1 [39], 2 [40] and 3 [41], respectively.


$$\mathrm{Mean}\;\mathrm{germination}\;\mathrm{time}=\frac{\sum_{i=1}^{k}n_{i}t_{i}}{\sum_{i=1}^{k}n_{i}}$$ Eq 1

Here, n_i_ti = The product of seeds germinated at interval i^th^ with the corresponding time interval, n_i_ = number of seeds germinated in the i^th^ time.


$$\mathrm{Time}\;\mathrm{to}\;\mathrm{reach}\;50\%\;\mathrm{germination}=\frac{t_{i}+(\frac{\sum_{i=1}^{k}n_{i}‐n_{i}}{2})(t_{j}‐t_{i})}{n_{j}‐n_{i}}$$ Eq 2

$$\mathrm{Mean}\;\mathrm{daily}\;\mathrm{germination}=\frac{\mathrm{Cummulative}\;\mathrm{germination}}{\mathrm{Number}\;\mathrm{of}\;\mathrm{days}\;\mathrm{taken}\;\mathrm{to}\;\mathrm{cummulative}\;\mathrm{germination}}$$ Eq 3

RETRACTED

### Statistical analysis

Differences in seed germination indices of two experimental runs were tested first with paired t test. The differences among two sets of same experiment were non-significant. Therefore, data of both experiments for a given environmental cue were pooled. Shapiro-Wilk normality test was used to infer the distribution of the data [42], and data were normally distributed. Hence original data were used for statistical analysis. The data were analyzed by Analysis of Variance (ANOVA) technique [43]. Two-way ANOVA was performed for testing significance. Least significant difference (LSD) post-hoc test at 5% probability was used to compare the means where ANOVA described significant differences. The results of ANOVA are given in S1 File.

## Results

Seed germination percentage and mean daily germination (MDG) significantly altered by individual and interactive effects of populations and light/dark periods. Mean germination time (MGT) and time to reach 50% germination (T_50_) were only affected by interactive effect of populations and light/dark periods (S1 File).

The lowest number of days were taken by temperate population for MGT under 12 hours light/dark period, while all remaining populations took higher number of days for MGT under the same light/dark regime. Seeds of temperate population took lesser number of days for T_50_ under 12 hours light/dark period, whereas arid populations took the highest number of days for MGT under same light/dark regime (Table 3). Similarly, semi-arid population under 0/24 light dark period recorded the lowest MDG, whereas the highest MDG was observed for the same population under 12 hours light/dark period (Table 3).

RETRACTED

**Table 3:** The impact of different light/dark durations on various germination indices of *Conyza sumatrensis* populations collected from varying climatic regions.

Populations	Light/dark periods		
	0L/24D	12L/12D	24L/0D
**Mean emergence time (days)**			
**Arid**	6.90 abc	7.34 c	6.39 ab
**Semi-arid**	6.68 abc	7.42 c	6.96 abc
**Humid**	7.13 bc	7.37 c	6.47 ab
**Temperate**	6.86 abc	6.28 a	6.91 abc
**LSD 5%**	0.74		
**Time to 50% emergence (days)**			
**Arid**	6.50 bcde	6.91 de	5.94 abc
**Semi-arid**	6.19 abcd	6.74 cde	6.49 bcde
**Humid**	6.63 bcde	7.26 e	5.94 ab
**Temperate**	6.33 abcd	5.68 a	6.55 bcde
**LSD 5%**	0.80		
**Mean daily germination (seeds day** ^**-1**^ **)**			
**Arid**	1.14 ab	5.66 e	2.28 c
**Semi-arid**	0.85 a	6.57 g	3.19 d
**Humid**	1.04 ab	5.81 ef	2.47 c
**Temperate**	1.33 b	6.00 f	2.23 c
**LSD 5%**	0.29		

Means followed by same letters within a column or row are statistically similar (p > 0.05) for the respective germination indices, 0 L = 0 hours light period, 24D = 24 hours dark period, 12L = 12 hours light period, 12D = 12 hours dark period, 24L = 24 hours light period, 0D = 0 hours dark period.

Different light/dark periods had significant effect on seed germination of different populations studied with the highest seed germination observed under 12 hours light and 12 hours dark period for all populations (Fig 1).

**Fig 1:** Seed germination percentage of different *Conyza sumatrensis* populations stemming from various climatic regions under different light and dark periods.

Individual and interactive effects of populations and different constant temperatures significantly affected seed germination percentage and MDG. The MGT and T_50_ were only affected by interactive effect of populations and constant temperatures, whereas their individual effects remained non-significant in this regard (S1 File).

Semi-arid and arid populations took the lowest number of days for MGT under 25°C, while arid population under 35°C took the highest number of days for MGT (Table 4). Semi-arid and arid populations took the highest and the lowest number of days for T_50_ under 30°C and 25°C constant temperature, respectively (Table 4). Likewise, semi-arid and arid populations observed the highest MDG under 25°C, while the lowest MDG was noted for semi-arid and humid populations under 5°C constant temperature (Table 4).

**Table 4:** The impact of different constant temperatures on various germination indices of *Conyza sumatrensis* populations collected from varying climatic regions.

Constant Temperatures	Populations			
	Arid	Semi-arid	Humid	Temperate
**Mean germination time (days)**				
**5°C**	7.73 a-f	8.16 a-c	8.13 abc	7.84 a-f
**10°C**	7.59 a-g	7.98 a-f	8.00 a-e	7.17 fgh
**15°C**	7.55 b-g	7.28 d-h	6.91 ghi	7.37 c-h
**20°C**	6.62 h-j	6.34 i-k	6.63 hij	7.20 e-h
**25°C**	5.49 l	5.52 l	5.73 kl	5.85 jkl
**30°C**	8.22 ab	8.28 ab	8.10 abc	7.83 a-f
**35°C**	8.37 a	8.08 a-d	7.98 a-f	8.05 a-d
**LSD 5%**	0.81			
**Time to 50% germination (days)**				
**5°C**	7.15 a-e	7.66 ab	7.69 ab	7.33 a-d
**10°C**	7.00 b-f	7.58 abc	7.40 a-d	6.60 d-h
**15°C**	6.95 b-g	6.70 d-h	6.32 e-h	6.72 c-h
**20°C**	6.09 ghi	5.87 hij	6.18 fgh	6.60 d-h
**25°C**	4.85 k	4.91 k	5.18 jk	5.25 ijk
**30°C**	7.99 a	7.98 a	7.65 ab	7.43 a-d
**35°C**	7.77 ab	7.65 ab	7.32 abcd	7.44 a-d
**LSD 5%**	0.87			
**Mean daily germination (seeds day** ^**-1**^ **)**				
**5°C**	1.00 kl	0.38 m	0.57 m	0.90 l
**10°C**	1.23 jk	1.00 kl	1.28 j	1.28 j
**15°C**	3.85 f	3.28 g	3.85 f	3.28 g
**20°C**	5.85 c	6.28 ab	5.66 c	4.71 d
**25°C**	6.42 ab	6.52 a	6.19 b	6.42 ab
**30°C**	4.14 e	3.38 g	2.28 h	1.57 i
**35°C**	1.57 i	1.33 ij	1.57 i	1.28 j
**LSD 5%**	0.26			

Means followed by same letters within a column or row are statistically similar (p > 0.05) for the respective germination indices.

RETRACTED

Individual and interactive effects of populations and different alternating temperatures significantly altered all seed germination indices of seeds collected from different climatic regions (S1 File).

Semi-arid population took the lowest number of days for MGT under 15°C /15°C, while arid population under same alternating temperature regime took the highest number of days for MGT (Table 5). Arid population under 20°C /10°C and semi-arid and humid populations under 20°C /15°C took lowest number of days T_50_ (Table 5). Likewise, semi-arid populations under 20°C/15°C observed the highest mean daily germination, whereas all population except semi-arid recorded the lowest MDG under 15°C /10°C (Table 5).

**Table 5:** The impact of different alternating day/night temperatures on various germination indices of *Conyza sumatrensis* populations collected from varying climatic regions.

Alternating Temperatures	Populations			
	Arid	Semi-arid	Humid	Temperate
**Mean germination time (days)**				
**15°C /10°C**	7.55 c	7.01 def	7.53 c	5.61 h
**15°C /15°C**	8.48 a	6.78 f	6.89 def	8.08 b
**20°C /10°C**	6.13 g	6.82 ef	7.17 cde	8.07 b
**20°C /15°C**	6.87 def	5.89 gh	5.94 gh	7.24 cd
**LSD 5%**	0.39			
**Time to 50% germination (days)**				
**15°C /10°C**	7.13 b	6.66 cde	7.07 bc	5.20 f
**15°C /15°C**	8.07 a	6.31 e	6.51 de	7.74 a
**20°C /10°C**	5.55 f	6.28 e	6.65 cde	7.95 a
**20°C /15°C**	6.56 de	5.46 f	5.55 f	6.85 bcd
**LSD 5%**	0.45			
**Mean daily germination (seeds day** ^**-1**^ **)**				
**15°C /10°C**	4.00 h	4.71 f	4.00 h	3.85 h
**15°C /15°C**	5.42 e	6.00 c	5.42 e	4.42 g
**20°C /10°C**	5.85 cd	5.28 e	5.42 e	4.28 g
**20°C /15°C**	6.28 b	6.57 a	5.71 d	4.85 f
**LSD 5%**	0.24			

Means followed by same letters within a column or row are statistically similar (p > 0.05) for the respective germination indices.

RETRACTED

Constant and alternating temperature significantly altered seed germination of population stemming from various climatic regions in the current study. Seeds of the population arising from arid and semi-arid region proved more resistant to increasing temperature compared to those stemming from temperate and humid regions (Figs 2 and 3). Overall, all populations observed the peak seed germination at same temperature, i.e., 25°C. However, seed of arid and semi-arid populations exhibited higher seed germination under higher temperatures as well where seeds of other populations were unable to germinate.

**Fig 2:** Seed germination percentage of different *Conyza sumatrensis* populations collected from various climatic regions under different constant temperatures.

**Fig 3:** Seed germination percentage of different *Conyza sumatrensis* populations collected from various climatic regions under different fluctuating day/night temperatures.

Individual and interactive effects of populations and different salinity levels significantly altered all seed germination indices (S1 File).

Semi-arid population under 0 and 400 mM salinity tool the lowest and highest number of days for MGT (Table 6). Temperate population under 350 mM salinity took the highest number of days for T_50_, whereas all populations reached T50 earlier under 0 mM salinity (Table 6). Likewise, all populations observed the highest mean daily germination under 0 mM salinity, whereas all population recorded the lowest MDG under 500 mM salinity (Table 6).

**Table 6:** The impact of different salinity levels on various germination indices of *Conyza sumatrensis* populations collected from varying climatic regions.

Salinity levels (mM NaCl)	Populations			
	Arid	Semi-arid	Humid	Temperate
**Mean germination time (days)**				
**0**	6.07 mno	5.43 o	5.59 no	6.28 mno
**25**	6.88 klm	6.76 lm	6.96 j-m	7.30 jkl
**50**	6.78 lm	6.31 l-no	6.53 lmn	7.79 ijk
**100**	9.17 fgh	9.17 fgh	9.42 fgh	9.88 d-g
**150**	9.04 gh	9.48 fg	10.10 c-f	9.09 gh
**200**	9.88 d-g	9.29 fgh	10.63 b-e	9.08 gh
**250**	9.28 fgh	9.52 fg	11.26 b	10.70 bcd
**300**	9.65 efg	10.16 c-f	10.94 bc	10.14 c-f
**350**	9.91 d-g	10.85 bcd	7.91 ij	8.43 hi
**400**	9.54 fg	12.34 a	0.00 p	0.00 p
**450**	6.50 lmn	9.01 gh	0.00 p	0.00 p
**500**	0.00 p	0.00 p	0.00 p	0.00 p
**LSD 5%**	1.00			
**Time to 50% germination (days)**				
**0**	5.48 jk	4.92 k	5.01 k	5.37 jk
**25**	6.34 jk	6.53 jk	6.40 jk	6.48 jk
**50**	6.35 jk	5.89 jk	5.82 jk	7.14 j
**100**	9.16 hi	9.16 hi	9.09 i	9.67 ghi
**150**	9.78 f-i	9.45 ghi	10.09 e-i	10.43 d-i
**200**	9.95 e-i	9.09 i	10.39 d-i	9.05 i
**250**	10.20 d-i	9.06 i	10.63 c-i	10.48 c-i
**300**	11.16 c-g	9.74 f-i	11.54 b-f	12.29 abc
**350**	11.98 a-d	10.40 d-i	11.16 c-g	13.38 a
**400**	13.20 ab	11.70 a-e	0.00 l	0.00 l
**450**	10.95 c-h	11.00 c-fg	0.00 l	0.00 l
**500**	0.00 l	0.00 l	0.00 l	0.00 l
**LSD 5%**	1.83			
**Mean daily germination (seeds day** ^**-1**^ **)**				
**0**	6.47 a	6.47 a	6.42 a	6.42 a
**25**	6.14 bc	6.28 ab	5.85 de	6.00 cd
**50**	5.85 de	5.71 ef	5.28 hi	5.57 fg
**100**	5.42 gh	5.42 gh	4.28 k	4.71 j
**150**	5.09 i	4.71 j	3.85 m	4.14 kl
**200**	4.71 j	4.28 k	3.28 n	3.85 m
**250**	4.28 k	3.85 m	2.85 p	3.14 no
**300**	4.00 lm	3.14 no	1.71 r	2.42 q
**350**	3.00 op	2.28 q	0.71 st	1.71 r
**400**	2.42 q	1.61 r	0.00 u	0.00 u
**450**	1.71 r	0.85 s	0.00 u	0.00 u
**500**	0.85 s	0.52 t	0.00 u	0.00 u
**LSD 5%**	0.21			

Means followed by same letters within a column or row are statistically similar (p > 0.05) for the respective germination indices.

RETRACTED

Individual and interactive effects of populations and different osmotic potential levels significantly altered seed germination percentage of seeds collected from different climatic regions (S1 File). Increasing salinity and osmotic potential suppressed seed germination of all populations; however, a lower decline was observed in the seed gemination of arid and semi-arid populations compared to humid and temperate populations (Figs 4 and 5). Seeds of arid and semi-arid populations germinated under higher salinity and osmotic potential compared to the seeds of humid and temperate populations.

**Fig 4:** Seed germination percentage of different *Conyza sumatrensis* populations collected from various climatic regions under different salinity stress levels.

**Fig 5:** Seed germination percentage of different *Conyza sumatrensis* populations collected from various climatic regions under different osmotic stress levels.

Individual and interactive effects of populations and different pH levels significantly altered seed germination percentage of seeds collected from different climatic regions (S1 File). Seed germination of different populations collected from various climatic regions was significantly altered by varying pH levels. However, a lower decline was observed in the seed gemination of arid and semi-arid populations compared to humid and temperate populations under higher pH (Fig 6). Seeds of arid and semi-arid populations germinated under higher pH compared to the seeds of humid and temperate populations.

**Fig 6:** Seed germination percentage of different *Conyza sumatrensis* populations collected from various climatic regions under different pH levels.

RETRACTED

Individual and interactive effects of populations and different seed burial depths significantly altered all seedling emergence percentage of seeds collected from different climatic regions (S1 File). Seedling emergence of different populations collected from varying climatic regions differed among various seed burial depths. Increasing depth of burial initially stimulated emergence up to 2 cm and then emergence percentage recorded a steep decline (Fig 7).

**Fig 7:** Seedling emergence percentage of different *Conyza sumatrensis* populations collected from various climatic regions under different seed burial depths.

## Discussion

Different environmental cues and their levels significantly altered seed germination indices of different *C*. *sumatrensis* populations collected from different climatic regions (S1 File). This supported our hypothesis that seed germination of different populations will significantly differ. The differences in populations are direct effect of the environmental cues faced by the maternal plants. Plenty of literature is available that supports our results pertaining to differences among seed germination biology of different populations due to maternal environments [14, 15, 17, 18, 44]. However, genetic factors also mediate the germination traits of different populations. Unfortunately, no such data is available to support our hypothesis, and this should be explored in future studies.

Our second hypothesis pertaining to the impacts of environmental cues on seed germination biology of the studied populations also stood valid and there are plenty of evidences to support our hypothesis [13–15, 17, 18, 45]. Seeds of *Conyza* species require a definite light period for their successful seed germination. This photoblastic behavior of the seeds has been described in several earlier studies.

Little differences were noted in the populations and population stemming from semi-arid region recorded the highest seed germination. The differences can be linked to the maternal impacts as semi-arid regions are rarely tilled and seeds remain near the soil surface. Thus, the seeds deposited in the soil surface have evolved to respond to light more compared to the seeds which are buried deep in the soil. The photoblastic nature of *Conyza* species has been reported in several earlier studies [26, 27, 46, 47].

Temperature is responsible for the activation of several necessary enzymes required to initiate seed germination [20]. Since the studied species is a winter annual, the decreased seed germination under high temperature can be explained with the nature of the species [8, 48]. Differences among populations are linked with the maternal effects as semi-arid and arid populations have undergone harsh environmental conditions; thus, became able to germanite under a wide range of environmental conditions.

RETRACTED

Salinity and drought are the most influential environmental cues negatively impacting seed germination of weed species [49]. However, weeds species possess various traits to cope salinity and drought to persist under harsh environmental conditions [49–51]. Soil salinity and temperature prevailing at the sites of seed collection is responsible of the differences in seed germination potential of tested populations in the current study. The differences in salinity and drought tolerance of different populations have been explained in earlier studies [13, 15].

Water imbibition of seeds is strongly altered by the pH of the soil. Neutral pH results in the optimum imbibition, whereas any deviation from this pH level results in disturbed water relations of the seeds [13, 20, 52, 53]. The decreased seed germination under higher pH is the result of lower water uptake. The differences among populations are due to maternal effects and soil properties of the seed collection sites.

The depth of burial has strong impact on water imbibition and contact of the soil with seed. Nevertheless, light penetration is also influenced by the seed burial depth. The deep-buried seeds are unable to perceive the required light intensity/duration required for seed germination, whereas the seeds placed on the surface loose moisture readily. Therefore, shallow, and deep burial both suppressed seedling emergence. Since seeds of all population required a definite light period for successful seed germination, deep burial-induced reduced seedling emergence can be explained with the absence of necessary light period required for seedling emergence. The amount of soil over the deep-buried seed also offers resistance in the emergence, which can also be a reason of decreased emergence. Deep burial-induced reduced seedling emergence of several *Conyza* species has been reported in earlier studies [18, 20, 52–54].

## Conclusion

Different populations arising from varying climatic regions significantly differed for their seed germination potential and seeds of arid and semi-arid populations had higher germination ability even under harsher environmental cues. Light was a necessary factor for the germination and 12-hour light period was necessary to induce seed germination. Higher temperature, salinity and osmotic stress levels suppressed germination of seeds collected from temperate and humid regions, whereas the seeds of arid and semi-arid regions exhibited higher germination ability under increased temperature, salinity, and osmotic stress levels. Seedling emergence was reduced beyond 2 cm burial depth indicating that deep seed burial followed by reduced or zero tillage could be a pragmatic approach to manage the species.

RETRACTED

## Supporting information

S1 File Analysis of variance tables for germination indices of *Conyza sumatrensis* populations collected from different climatic regions under various environmental cues. (DOCX)
